This article has been retracted.

# Rosiglitazone Exerts an Anti-depressive Effect in Unpredictable Chronic Mild-Stress-Induced Depressive Mice by Maintaining Essential Neuron Autophagy and Inhibiting Excessive Astrocytic Apoptosis

**DOI:** 10.3389/fnmol.2017.00293

**Published:** 2017-09-14

**Authors:** Zhan Zhao, Ling Zhang, Xu-Dong Guo, Lu-Lu Cao, Teng-Fei Xue, Xiao-Jie Zhao, Dan-Dan Yang, Jin Yang, Juan Ji, Ji-Ye Huang, Xiu-Lan Sun

**Affiliations:** ^1^Neuroprotective Drug Discovery Key Laboratory, Department of Pharmacology, Nanjing Medical University Nanjing, China; ^2^Neuroprotective Drug Discovery Key Laboratory, Department of Forensic Medicine, Nanjing Medical University Nanjing, China

**Keywords:** PPARγ, rosiglitazone, depression, neuron, astrocyte, autophagy, apoptosis

## Abstract

There is increasing interest in the association between depression and the development of metabolic diseases. Rosiglitazone, a therapeutic drug used to treat type 2 diabetes mellitus, has shown neuroprotective effects in patients with stroke and Alzheimer’s disease. The present study was performed to evaluate the possible roles of rosiglitazone in *in vivo* (unpredictable chronic mild stress-induced depressive mouse model) and *in vitro* (corticosterone-induced cellular model) depressive models. The results showed that rosiglitazone reversed depressive behaviors in mice, as indicated by the forced swimming test and open field test. Rosiglitazone was also found to inhibit the inflammatory response, decrease corticosterone levels, and promote astrocyte proliferation and neuronal axon plasticity in the prefrontal cortex of mice. This series of *in vivo* and *in vitro* experiments showed that autophagy among neurons was inhibited in depressive models and that rosiglitazone promoted autophagy by upregulating LKB1, which exerted neuroprotective effects. Rosiglitazone was also found to activate the Akt/CREB pathway by increasing IGF-1R expression and IGF-1 protein levels, thereby playing an anti-apoptotic role in astrocytes. Rosiglitazone’s autophagy promotion and neuroprotective effects were found to be reversed by the PPARγ antagonist T0070907 in primary neurons and by PPARγ knockdown in an N2a cell line. In conclusion, we found that rosiglitazone protects both neurons and astrocytes in *in vivo* and *in vitro* depressive models, thereby playing an anti-depressive role. These findings suggest that PPARγ could be a new target in the development of anti-depressive drugs.

## Introduction

Over the past few decades, depression has become one of the most common neuropsychiatric disorders, affecting the quality of life of millions of people worldwide (Kessler et al., 2003). The WHO estimates that by 2020, depression may become the second largest contributor to disability. Numerous studies have demonstrated that the etiology of depression includes not only stress-induced mental issues but also stress-induced pathological lesions, particularly in encephalic regions (Krishnan and Nestler, 2008), and especially in the prefrontal cortex (PFC) and hippocampus, although the underlying mechanism remains largely unknown. Generally, patients with depression exhibit depressive behavior and specific pathological symptoms such as deficiencies of cell proliferation and neuroplasticity, inflammatory responses, and abnormal cytokine secretion (Snyder et al., 2011; Sarkar et al., 2014; Walker et al., 2014; Malykhin and Coupland, 2015; Henry et al., 2016). Unpredictable chronic mild stress (UCMS) is widely used to produce depressive animal models because it can lead to depressive behavior in rodents (Voorhees et al., 2013). It is widely recognized that chronic stress causes the release of glucocorticoids and corticosterone in humans and rodents (Barik et al., 2013; McEwen, 2013; Niwa et al., 2013), and depression is accompanied by the secretion of high levels of corticosterone. High levels of glucocorticoids and corticosterone may affect multiple physiological reactions related to depression in neurons and astrocytes, such as apoptosis, autophagy, and synaptic plasticity (He et al., 2016; Zeng et al., 2016; Chen et al., 2017). Treating neurons and glial cells with corticosterone is often used to establish *in vitro* depressive models.

While exploring new therapeutic strategies for dealing with depression, numerous groups have focused on the anti-depressive role of certain antidiabetic agents, attributed to the fact that there is a strong association between depression and metabolic syndrome, especially type 2 diabetes mellitus (Golden et al., 2008; Igna et al., 2011; Kahl et al., 2015). Approximately 25% of individuals with diabetes exhibit depressive symptoms, and diabetes appears to be a risk factor for depression (Goldney et al., 2004; Nouwen et al., 2010). In such cases, many kinds of antidiabetic agents, such as metformin, sulfonylureas, and thiazolidinediones, have been confirmed or inferred to relieve depression (Biemans et al., 2015; Sheikh et al., 2015; Colle et al., 2017b).

Rosiglitazone, a thiazolidinedione drug widely used as an insulin-sensitizing agent to relieve type 2 diabetes mellitus, has been reported to exert neuroprotective effects in several conditions affecting the central nervous system (Yki-Jarvinen, 2004), such as Parkinson’s disease (PD) (Normando et al., 2016; Pinto et al., 2016), Alzheimer’s disease (AD) (Bonet-Costa et al., 2016; Vallee and Lecarpentier, 2016), and stroke (Certo et al., 2015; Liu and Wang, 2015; Xiong et al., 2016). Notably, pioglitazone, which has a chemical structure similar to that of rosiglitazone, was found to relieve depression (Colle et al., 2017a; Liao et al., 2017), and Patel et al. (2015) reported that rosiglitazone was also effective in the treatment of neurological disorders associated with depression-like behavior. As the specific target of rosiglitazone, peroxisome proliferator-activated receptor γ (PPARγ) was found to be downregulated in the neurons of mice that exhibited depression-like behavior (Zhou et al., 2014), and PPARγ agonists (including rosiglitazone) were found to be effective antidepressants in both rodents and humans (Colle et al., 2017b). However, the details underlying these mechanisms remain unknown.

In the present study, the therapeutic effect of rosiglitazone was observed in a UCMS-induced depressive mouse model and corticosterone-induced depressive cellular model. The results showed that rosiglitazone exerted anti-depressive effects by maintaining essential autophagy in neurons and protecting astrocytic apoptosis in the prefrontal cortexes of mice.

## Materials and Methods

### Experimental Animals and Procedures

Seven- to 8-week-old male C57BL/6 mice weighing 25 ± 2 g were obtained from the Animal Resource Center of the Faculty of Medicine, Nanjing Medical University for use in the experiment. All mice were kept in a standardized environment (temperature 25 ± 2°C, humidity 55 ± 10%, irradiation time 8:00–20:00) and single-housed in the Animal Resource Centre of the Faculty of Medicine, Nanjing Medical University. The entire experimental process and animal treatment adhered to the rules of the Experimental Animal Application Criteria and Institutional Animal Care and Use Committee (IACUC). All of the experimental mice were allowed to adapt to the new environment for 1 week before the experiment. After three times of the sucrose preference test (SPT), mice were divided into the control group and UCMS group according to the results of the SPT and their weights. After 6 weeks of UCMS exposure, UCMS group mice were divided into UCMS control group, fluoxetine-treated UCMS group (10 mg/kg), and rosiglitazone-treated UCMS group (5 mg/kg, 0.1 M hydrochloric acid used as the dissolution medium). Afterward, intraperitoneal injections were administered for another 6 weeks in each group.

### Sucrose Preference Test

Mice were deprived of water for 12 h before SPT. Then, two drinking bottles containing 1% sucrose water or sterile water were placed in the drinking hole of each cage. The sites of the drinking bottles were switched 6 h later to preclude the influence of drinking site preference. After another 6 h, the regular water supply was restored and both bottles were weighed. The change in weight of each bottle equaled the sucrose water or sterile water intake. The SPT value was then calculated using the following formula:

SPT(%)=sucrose⁢ water⁢ intake/(sucrose⁢ water⁢ intake+ sterile⁢ water⁢ intake)×100%.

### Unpredictable Chronic Mild Stress

Unpredictable chronic mild stress is known to be an effective method for inducing depression-like behavior. To create a UCMS model, we exposed the experimental mice to a number of stressors, including a 45° sloped cage (6 h), a wet cage (200 ml sterile water added to the cage; 6 h), restrained motion (shut mice in a brown glass bottle with 3 cm radius and 15 cm height for 2 h), pairing (placed two unfamiliar mice in a cage for 2 h), food and water deprivation (24 h, avoiding the SPT days), switched day/night lights, and tail clamping (20 min). The mice received two or three random stressors daily to ensure unpredictability.

### Forced Swimming Test (FST)

The forced swimming test is a common method for evaluating depression-like behavior. After 12 weeks of UCMS modeling or administration, the FST was carried out in all four groups of mice. Mice were individually placed in 2 L beakers containing 1 L of water at 25°C. A camera recorded the movement of the mice for 6 min. Subsequently, the video was analyzed by Tail Suspension Scan (Clever Sys Inc., Reston, VA, United States). Escape time was defined as the time during which the mouse’s legs or body moved.

### Open Field Test (OFT)

The open field test is commonly used to evaluate locomotor activity and spontaneous exploration in a novel environment. Activity monitoring was conducted in a square area measuring 40 cm × 40 cm × 30 cm. The center area was defined as a square 10 cm away from the wall. The total duration in the center was recorded as an index of anxiety. Mice were placed individually into the periphery of the area and allowed to explore freely for 5 min while being monitored with a video camera. The data were analyzed using the Open Field Scan (Clever Sys Inc., Reston, VA, United States).

### Cell Culture and Treatment

Primary cortex astrocyte and neuron cultures were created as previously described (Shan et al., 2016). The neurons and astrocytes were treated with various reagents: corticosterone (Sigma, United States), rosiglitazone (dissolved in dimethyl sulfoxide [DMSO] to ≤0.1% v/v; MedChemExpress, United States), 10 μM PPARγ inhibitor T0070907 (Selleck, China), 10 μM Akt inhibitor LY294002 (Sigma, United States), 10 μM AICAR (Sigma, United States), 1 μM compound C (Sigma, United States). Additionally, astrocytes were treated with 5 nM recombinant IGF-1 (Abcam, United States). After exposure to 1 ml DMEM-supplemented corticosterone or rosiglitazone for 24 h, the medium was collected and used as conditional medium in the neuron culture for further corticosterone or rosiglitazone treatment.

### Cell Transfection

N2a cells were placed in 6-well plates at 4 × 10^5^ cells per well overnight. Then the plasmid (Mock: P3XFLAG-CMV7.1) and *PPARγ-mus*-siRNA (GenePharma, Shanghai, China; sequence: GCGGAGAUCUCCAGUGAUATT; UAUCACUGGAGAUCUCCGCTT) were transfected for 6 and 8 h, respectively, using Lipofectamine 2000 (Invitrogen, United States), according to the manufacturer’s instructions.

### Lactate Dehydrogenase Assay and MTT

Cells were placed in 96-well plates at a density of 1 × 10^4^ cells per well for 24 h before corticosterone stimulation or treatment. Supernatants were collected, and the concentration of LDH was detected using an assay kit (Jiancheng Bioengineering Institute, Nanjing, China). MTT (0.5 mg/ml) was dissolved in the cell medium and incubated at 37°C for 4 h. Then, DMSO was used to dissolve the MTT-formazan product. All absorbance was obtained using a Dynatech MR5000 plate counter at a test wavelength of 570 nm.

### Serum Sampling for Enzyme-Linked Immunosorbent Assay (ELISA)

Serum samples were obtained by the retro-orbital bleeding assay and then clotted overnight at 4°C before centrifugation for 20 min at 1000 × *g*. The concentration of IL-6, TNFα, corticosterone, IGF-1, VEGF, and CNTF in the serum was detected by an ELISA kit (Cloud Clone Corp., United States) according to the manufacturer’s instructions.

### Quantitative Reverse Transcription-Polymerase Chain Reaction (qRT-PCR)

Total RNA was isolated from brain tissues, cell samples, or cultured cells using TRIzol reagent (Karroten) and prepared for quantitative reverse transcriptase PCR using Master Mix (TaKaRa, Japan). Primer sequences were designed by Primer Premier 6 as **Table 1**. Real-time PCR was carried out using the SYBR Green mixture (TaKaRa, Japan) in a QuantStudio 5 system (Thermo Fisher Scientific, United States). The cycling conditions were as follows: denaturation at 95°C for 30 s, followed by 40 cycles of DNA synthesis at 95°C for 5 s and 60°C for 34 s. All results were measured using the 2^-ΔΔCT^ method.

**Table 1:** Primer sequences.

*Gene*	Accession	Sense	Antisense
*il-1*β	NM_008361.4	GAAATGCCACCTTTTGACAGTG	TGGATGCTCTCATCAGGACAG
*il-6*	NM_001314054.1	CTGCAAGAGACTTCCATCCAG	AGTGGTATAGACAGGTCTGTTGG
*il-10*	NM_010548.2	CTTACTGACTGGCATGAGGATCA	GCAGCTCTAGGAGCATGTGG
*tnf*α	NM_001278601.1	CAGGCGGTGCCTATGTCTC	CGATCACCCCGAAGTTCAGTAG
*inos*	NM_001313922.1	AACAGAGCCCTCAGCAGCATCCAT	CCAGGTGTTCCCCAGGCAGGTAG
*mmp9*	NM_013599.4	GCAGAGGCATACTTGTACCG	TGATGTTATGATGGTCCCACTTG
*bdnf*	NM_001316310.1	TCATACTTCGGTTGCATGAAGG	ACACCTGGGTAGGCCAAGTT
*gdnf*	NM_001301357.1	GCCGGACGGGACTCTAAGAT	CGTCATCAAACTGGTCAGGATAA
*vegf*	NC_000083.6	CTGCCGTCCGATTGAGACC	CCCCTCCTTGTACCACTGTC
*cntf*	NM_170786.2	TCTGTAGCCGCTCTATCTGG	GGTACACCATCCACTGAGTCAA
*nt3*	NM_001164035.1	AGTTTGCCGGAAGACTCTCTC	GGGTGCTCTGGTAATTTTCCTTA
*ngf*	NM_013609.3	TGATCGGCGTACAGGCAGA	GCTGAAGTTTAGTCCAGTGGG
*igf1*	NM_010512.5	CACATCATGTCGTCTTCACACC	GGAAGCAACACTCATCCACAATG
*ppar*γ	NM_001308354.1	GGAAGACCACTCGCATTCCTT	GTAATCAGCAACCATTGGGTCA
*cab39*	NM_133781.4	CCGTTCCCATTTGGCAAGTCT	TCATTGGTGCCGTACAGAATTTC
*strad*	NM_028126.3	AGAGGGCGGGTGTTATGAG	GGTTGATCCTTCGTACTGTCAC
*gapdh*	NM_001289726.1	CATGGCCTTCCGTGTTCCTA	CCTGCTTCACCACCTTCTTGAT

The prefrontal cortexes or cell samples were disintegrated in a lysis buffer consisting of 1% PMSF. A BCA Kit (KeyGEN BioTECH, China) was used to measure the concentration of each protein sample. Then, the proteins were separated on 8–12% SDS-polyacrylamide gels and transferred onto methyl alcohol-soaked PVDF membranes (Millipore, United States). After blocking in 10 mM Tris buffer containing 0.2% Tween-20 (TBST) and 5% non-fat milk at room temperature for 1 h, the membranes were incubated with specific primary antibodies (see **Table 1**) at 4°C overnight. After washing with TBST, membranes were incubated with HRP-conjugated secondary antibody (dilution 1:8000; Beyotime, China). After additional washing with TBST four times, protein bands were visualized by enhanced chemiluminescence (Tanon, China). The protein expression level of each sample was normalized to the gray value of GAPDH and analyzed by ImageJ software.

### Immunofluorescence

Sections of the brain were incubated in 3% H_2_O_2_ for 15 min to block endogenous peroxide and then washed with phosphate-buffered solution (PBS) three times. Next, sections were blocked with 5% goat serum and 0.01% Triton-100 (dissolved in PBS) for 1 h and then incubated with primary antibodies overnight at 4°C. Following washing with PBS, the sections were incubated with Alexa Fluor 488 or 555 donkey anti-mouse, anti-goat, or anti-rabbit secondary antibodies (1:1000 dilution, Invitrogen, United States). Images were captured by a fluorescence microscope (Olympus, Japan) after incubation in Hoechst 33258 (10 μg/ml, Sunshine Biotechnology, Nanjing, China) for 15 min and washing with PBS three times. All primary antibodies used are listed in **Table 2**.

**Table 2:** Primary antibodies.

Protein	Manufacture	Number	Dilution
CD11b	Abcam	ab1211	1:500


TNFα	Abcam	ab6671	1:400


GFAP	Millipore	MAB3402	1:200


NeuN	Millipore	MAB3402	1:200


Bcl2	Proteintech	12789-1-AP	1:1000


MAP2	Abcam	ab7756	1:200


Bax	Proteintech	23931-1-AP	1:1000
p-mTOR	Affbiotech	AF3308	1:500
mTOR	Proteintech	20657-1-AP	1:500
p-Akt	Cell Signaling Technology	4691	1:1000
Akt	Cell Signaling Technology	4060	1:1000
p-IRS1	Cell Signaling Technology	2388	1:500
IRS1	Abcam	ab52167	1:1000
LC3	Proteintech	14600-1-AP	1:1500
P62	Proteintech	18420-1-AP	1:1000
ULK1	Abcam	ab128859	1:1000


Beclin1	Proteintech	11306-1-AP	1:800
p-AMPK	Cell Signaling Technology	2535	1:1000
AMPK	Proteintech	18167-1-AP	1:1000


IGF1R	Abcam	ab39398	1:1000


Caspase 3	Cell Signaling Technology	9661	1:500
PARP	Abcam	ab32064	1:800
p-CREB	Cell Signaling Technology	9198	1:1000
CREB	Cell Signaling Technology	9197	1:1000
PPARγ	Proteintech	16643-1-AP	1:500
LKB1	Proteintech	10746-1-AP	1:1000
GAPDH	Proteintech	10494-1-AP	1:6000
H3	Proteintech	17168-1-AP	1:3000

### TdT dUTP Nick-End Labeling (TUNEL) Staining

Following the manufacturer’s instructions for the TUNEL kit (KeyGen Biotech, China), sections were incubated with proteinase K for 10 min, and TUNEL was performed for 1 h at 37°C. After washing with PBS three times, sections were incubated in Hoechst 33258 for 15 min. Finally, section images were captured by a fluorescence microscope.

### Flow Cytometry

Astrocyte samples were washed with PBS three times, then digested and centrifuged gently. Apoptotic cells were detected by flow cytometry (BD FACSCalibur, United States) after staining with an Annexin V-FITC/PI kit (KeyGen Biotech, China).

### Transmission Electron Microscope

Primary cortex neuron samples were collected by centrifugation and fixed with 3% glutaraldehyde overnight at 4°C and then fixed with 4% OsO_4_ at room temperature for 1 h. After gradient elution by acetone, samples were sliced into ultrathin sections and then observed with a transmission electron microscope (JEOL JEM-1010, Japan).

### Statistical Analysis

Statistical analyses were performed using GraphPad Prism 7. Multiple comparisons were conducted using one-way ANOVA, and Fisher’s least significant difference (LSD) test was used for *post hoc* comparisons. The means of the two treatment groups were analyzed using unpaired or paired Student’s *t*-tests. Data are expressed as means ± SEMs.

## Results

### Rosiglitazone Improves UCMS-Induced Depressive Behaviors

The experimental process shown in **Figure 1A** was established to validate the anti-depressive role of rosiglitazone. UCMS mice exhibited decreased sucrose preference and body weights compared with control group mice. Administration of fluoxetine and rosiglitazone ameliorated this effect (**Figures 1B,C**). To confirm these results, FST and OFT were performed to evaluate mouse behavioral despair and fear of new environments. After 6 weeks of UCMS and 6 weeks of rosiglitazone treatment, the UCMS-induced declines in escape time and center durations in FST and OFT disappeared (**Figures 1D,E**).

**FIGURE 1:** Antidepressant effects of rosiglitazone in unpredictable chronic mild stress (UCMS) mouse model. **(A)** Experimental process of UCMS modeling or administration. **(B)** SPT and **(C)** body weight changes of each group of mice. **(D)** The center and **(E)** escaping durations of mice in the OFT and FST. Data are presented as means ± SEMs, *n* = 10–16 for the behavior test. ^∗^*p* < 0.05 vs. control, ^∗∗∗^*p* < 0.001 vs. control, ^#^*p* < 0.05 vs. UCMS, ^##^*p* < 0.01 vs. UCMS, ^###^*p* < 0.001 vs. UCMS, ^$$^*p* < 0.01 vs. week 0 of UCMS group. UCMS+Flu, fluoxetine-treated UCMS group; UCMS+Rosi, rosiglitazone-treated UCMS.

### Rosiglitazone Ameliorates UCMS-Induced Neuron and Astrocyte Injury in the Prefrontal Cortex

A TUNEL assay was used to label apoptotic cells in tissue slices to determine whether rosiglitazone protected neural cells in the PFC. We found that the density of TUNEL-positive cells in the prelimbic cortex (PrL) of the PFC increased in UCMS mice, and this effect was ameliorated by rosiglitazone treatment (**Figures 2A,B**). Then, microtubule-associated protein 2 (MAP2), a marker specific to mature neurons, was used to stain neuronal somata and dendrites. The results showed that MAP2-labeled PFC neurons were shortened, and reduced axon length was observed in tissue slices from UCMS mice but not in the rosiglitazone administration groups (**Figure 2C**). Next, we labeled astrocytes with glial fibrillary acidic protein (GFAP), a widely used biomarker of astrocytes, and the results showed that rosiglitazone reversed UCMS-induced astrocyte reduction (**Figures 2D,E**). These data revealed that rosiglitazone mitigated UCMS-induced injuries to neurons and astrocytes in depressive mice.

**FIGURE 2:** Rosiglitazone protects astrocytes and neurons of UCMS mice in the PFC. **(A,B)** TUNEL-labeled apoptosis cells in rosiglitazone-group mice decreased compared with the UCMS group. **(C)** MAP2-positive neurons and axons in the PFC. **(D,E)** GFAP-positive astrocytes in mouse PFC sections. (I) Control. (II) UCMS. (III) UCMS + rosiglitazone. Data are presented as means ± SEMs, *n* = 5–6; ^∗∗^*p* < 0.01 vs. control, ^∗∗∗^*p* < 0.001 vs. control, ^#^*p* < 0.05 vs. UCMS. UCMS+Rosi, rosiglitazone-treated UCMS.

### Rosiglitazone Ameliorates the Inflammatory Response and Hormone/Cytokine Dysfunction

Because chronic inflammation is often associated with the development of symptoms of depression, the role of rosiglitazone in neuroinflammation in the prefrontal cortex was examined further. As shown in **Figure 3A**, UCMS mice exhibited higher levels of *IL-1*β, *IL-6*, and *TNF*α mRNA in the PFC and higher concentrations of IL-6 and TNFα in serum. These were significantly reduced by fluoxetine and rosiglitazone treatment (**Figures 3B,C**). Double-label immunofluorescence assays with TNFα and CD11b were used to detect microglia, the principal cells involved in the innate immune response in the central nervous system. The results showed that administration of rosiglitazone could inhibit UCMS-induced microglia activation (**Figures 3D,E**). These results indicate that rosiglitazone prevents UCMS-induced inflammatory responses.

**FIGURE 3:** Rosiglitazone influences inflammation, hormones, and cytokines of UCMS mice in the PFC or serum. **(A)** mRNA changes of inflammation-associated factors in the PFC. **(B,C)** The concentrations of IL-6 and TNFα detected by ELISA in serum. **(D,E)** Quantitative immunofluorescence analysis of TNFα-positive microglia in the PFC. **(F)** The concentrations of corticosterone in mouse serum. **(G)** mRNA levels of *BDNF*, *GDNF*,*VEGF*, *CNTF*, *NT3*, *NGF*, and *IGF-1* in the PFC as revealed by qRT-PCR. **(H–J)** The concentrations of CNTF, IGF-1, and VEGF detected by ELISA in serum. Data are presented as means ± SEMs; *n* = 5–6 for immunofluorescence and *n* = 8 for qRT-PCR and ELISA assays. ^∗^*p* < 0.05 vs. control, ^∗∗^*p* < 0.01 vs. control, ^∗∗∗^*p* < 0.001 vs. control, ^#^*p* < 0.05 vs. UCMS, ^##^*p* < 0.01 vs. UCMS, ^###^*p* < 0.001 vs. UCMS. UCMS+Flu, fluoxetine-treated UCMS group; UCMS+Rosi, rosiglitazone-treated UCMS.

Rosiglitazone also reduced UCMS-induced increases in the secretion of corticosterone, one hormone related to depression (**Figure 3F**). UCMS also downregulated mRNA levels of depression-related cytokines BDNF, GDNF, CNTF, and IGF-1 in the mouse PFC. Rosiglitazone increased the mRNA levels of *IGF-1* and *CNTF* (**Figure 3G**), and the ELISA assay showed similar results in mouse serum (**Figures 3H–J**).

### Rosiglitazone Upregulates Neuron Autophagy and Reduces Astrocyte Apoptosis in the Prefrontal Cortex

Autophagy has a crucial impact on cellular homeostasis, and it affects CNS diseases, including depression. The expression of ULK1, which acts as a convergence point for multiple signals that control autophagy, was lower in depressive mice than that in control mice. The decline in autophagy was followed by the downregulation of Beclin 1 and the LC3II/LC3I ratio along with upregulation of P62. AMP-activated protein kinase (AMPK) is an important upstream kinase of ULK1; its Thr 172-phosphorylated form also decreased in UCMS mice (**Figures 4C,D**). Rosiglitazone could upregulate the protein expression of LC3II, ULK1, Beclin 1, and p-AMPK and downregulate P62. Rosiglitazone could also increase the number of LC3B-labeled neurons (**Figures 4A,B**).

**FIGURE 4:** Autophagy- and apoptosis-related proteins are mediated by rosiglitazone administration. **(A)** Labeling of LC3B onto neurons in the sections and **(B)** counting the number of positive cells. **(C,D)** Analysis of autophagy-associated proteins LC3, P62, ULK1, Beclin 1, and p-AMPK/AMPK. **(E,F)** Western blotting analyzed the expression of Bcl2 Bax, and detected the ratio of p-mTOR, p-Akt and p-IRS1, GAPDH as a loading control. Data are presented as means ± SEMs; *n* = 5–6 for WB and *n* = 8–10 for IF. ^∗^*p* < 0.05 vs. control, ^∗∗^*p* < 0.01 vs. control, ^∗∗∗^*p* < 0.001 vs. control, ^#^*p* < 0.05 vs. UCMS, ^##^*p* < 0.01 vs. UCMS, ^###^*p* < 0.001 vs. UCMS. UCMS+Rosi, rosiglitazone-treated UCMS.

Furthermore, the effects of rosiglitazone on the expression of the pro-apoptotic protein BAX and the anti-apoptotic protein Bcl2 were detected by Western blotting. The Bcl2/BAX ratio declined markedly in response to UCMS and returned to normal after administration of rosiglitazone. Notably, rosiglitazone activated the Akt/mTOR pathway, which plays a vital role in cell survival, by phosphorylating Akt and mTOR at Ser 473 and Ser 2448, respectively. Rosiglitazone enhanced the phosphorylation of insulin receptor substrate 1 (IRS1, phosphorylated at Ser 636/639), which is considered to be the main activator of the Akt/mTOR pathway by IGF-1R (**Figures 4E,F**).

### Rosiglitazone Promotes Autophagy in Corticosterone-Treated Primary Neurons by Elevated Phosphorylation of AMPK

Exposure to 10 μM of corticosterone was found to significantly injure primary cultured cortex neurons (**Figure 5A**). Neurons exposed to 10 μM rosiglitazone released LDH less than those in the corticosterone groups (**Figure 5B**). Next, we observed the morphology and amount of LDH released from the neurons of the primary cortex and found that autophagy inhibitor 3-methyladenine (0.5 mM), which targets PI3K, reversed the protective effect of rosiglitazone (**Figures 5C,D**). Observing the intracellular autophagosomes by transmission electron microscopy is the most reliable method of confirming the presence of autophagy. We found that the amount of autophagosomes in primary neurons decreased after corticosterone exposure, whereas the autophagosomes in neurons treated with rosiglitazone increased markedly. Moreover, treatment with T0070907, an inhibitor of PPARγ, reversed this tendency (**Figure 5E**). Next, the expression of autophagy-related proteins was analyzed by Western blotting. The results indicated that corticosterone exposure could lead to the downregulation of LC3II/I, ULK1, and p-AMPK/AMPK and the upregulation of p-mTOR/mTOR and P62, which predicted the deficiency of autophagy. Rosiglitazone treatment was found to enhance the level of autophagy by reversing the changes induced by corticosterone, which was prevented by T0070907 (**Figures 5F,G**).

**FIGURE 5:** Corticosterone-induced autophagy deficiency in primary cortex neurons is relieved by rosiglitazone. **(A,B)** The vitality of neurons exposed to specific concentrations of corticosterone and rosiglitazone was measured by detecting LDH secretion. **(C)** Growth status of primary cortex neurons exposed to corticosterone, rosiglitazone, and T0070907 (10 μM) was observed using a transmission electron microscope. **(D)** LDH secretion assay showed that 3-MA (0.5 mM) was able to abolish the protective role of rosiglitazone in corticosterone-induced neuron injury. **(E)** Autophagosomes in primary neurons exposed to corticosterone, rosiglitazone, and T0070907 were observed using a transmission electron microscope. **(F–J)** Autophagy-related proteins LC3, ULK1, P62, p-mTOR, p-AMPK, and LKB1 were measured by WB in neurons exposed to an agonist or inhibitor of PPARγ and AMPK (AICAR: 10 μM, compound C: 1 μM). Data are presented as means ± SEMs; *n* = 4–6 for all groups. ^∗^*p* < 0.05 vs. control, ^∗∗^*p* < 0.01 vs. control, ^∗∗∗^*p* < 0.001 vs. control, ^#^*p* < 0.05 vs. corticosterone, ^##^*p* < 0.01 vs. corticosterone, ^###^*p* < 0.001 vs. corticosterone, ^$^*p* < 0.05 vs. cort+rosi, ^$$^*p* < 0.01 vs. cort+rosi, ^$$$^*p* < 0.001 vs. cort+rosi. cort, corticosterone; rosi, rosiglitazone; c+r, corticosterone + rosiglitazone; c+r+t, corticosterone + rosiglitazone+T0070907; c+r+CC, corticosterone + rosiglitazone + compound C; c+t+a, corticosterone + T0070907+AICAR.

To investigate the relationship between PPARγ and AMPK, pharmacological tools were used to treat neurons, and a Western blot assay was performed to assess the expression of related proteins. The results showed that compound C, an antagonist of AMPK, blocked the mitigation of the autophagic effects of rosiglitazone. In contrast, the AMPK agonist AICAR activated autophagy, even in the presence of T0070907 (**Figures 5H–J**). These results suggest that rosiglitazone maintains essential autophagy and protects cells from corticosterone-induced neuronal damage by elevating the phosphorylation of AMPK.

### Rosiglitazone Promotes Autophagy in Corticosterone-Treated N2a Cells via Activation of the LKB1/AMPK Pathway

In order to confirm the effects of rosiglitazone-mediated enhancement of autophagy via LKB1/AMPK pathway activation, PPARγ was knocked down or overexpressed in N2a cell lines. We found that rosiglitazone also protected N2a cells from corticosterone-induced decreases in cell viability (**Figures 6A,B**). Rosiglitazone protected N2a cells from corticosterone stimulation, and this effect could be reversed by 3-MA (**Figure 6C**). Notably, rosiglitazone failed to protect PPARγ-deficient N2a cells from corticosterone (**Figure 6D**). The results also showed that the expression of LKB1, an important AMPK upstream kinase, was increased by rosiglitazone, and this effect was reversed by T0070907 in N2a cells (**Figures 6E,F**). Taken together, these findings indicate that rosiglitazone prevents corticosterone-induced defects in autophagy in a PPARγ-dependent manner.

**FIGURE 6:** Rosiglitazone relieves corticosterone-induced N2a cell autophagy deficiency by enhancing autophagy via the LKB1/AMPK pathway. **(A,B)** The vitality of N2a cells exposed to specific concentrations of corticosterone and rosiglitazone was measured by the MTT assay. **(C)** Growth status of primary astrocytes exposed to (I) DMSO, (II) cort, (III) cort+rosiglitazone, (IV) cort+rosiglitazone+3-MA (0.5 mM). **(D)** Rosiglitazone was unable to relieve corticosterone-induced cell injury in *PPAR*γ-deficient N2a cells. **(E)** LKB1 and **(F)** p-AMPK/AMPK expressed in the N2a cell line. **(G)** *PPAR*γ, **(H)** *Mo25*, and **(I)** *STRAD* mRNA levels were increased or decreased when *PPAR*γ was knocked down or overexpressed. **(J–L)** The expressions of PPARγ and LKB1 proteins were increased or decreased when *PPAR*γ was knocked down or overexpressed. Data are presented as means ± SEMs; *n* = 4–6 for all groups. ^∗^*p* < 0.05 vs. control, ^∗∗^*p* < 0.01 vs. control, ^∗∗∗^*p* < 0.001 vs. control, ^#^*p* < 0.05 vs. corticosterone, ^##^*p* < 0.01 vs. corticosterone, ^$$^*p* < 0.01 vs. cort+rosi. cort, corticosterone; rosi, rosiglitazone; c+r, corticosterone + rosiglitazone; c+r+t, corticosterone + rosiglitazone+T007090.

Further, knockdown of *PPAR*γ by siRNA decreased the mRNA levels of *IKB-1* and its two accessory subunits, STE20-related adaptor protein (STRAD) and calcium-binding protein 39 (CAB39, also called Mo25), compared with the negative control group (NC). In contrast, overexpression of *PPAR*γ in the N2a cells upregulated *IKB-1*, *STRAD*, and *Mo25* (**Figures 6G–L**). These results suggest that rosiglitazone activates the LKB1/AMPK signal pathway to maintain essential autophagy and protect cells from corticosterone-induced neuronal damage.

### Rosiglitazone Inhibits Corticosterone-Induced Astrocyte Apoptosis by Upregulating IGF-1R and Activating the Akt/CREB Pathway

IGF-1 is mostly derived from the peripheral organs, such as the liver or spleen, via serum, although astrocytes can also secrete moderate amounts of IGF-1. Here, the primary astrocytes were cultured with DMEM and 5 nM recombinant mouse IGF-1 protein to determine the mechanisms involved in rosiglitazone-mediated protective effects. The results showed that rosiglitazone protected astrocytes from corticosterone-induced injury to a significant extent (**Figures 7A,B**), and Hoechst staining of primary astrocytes showed that T0070907 inhibited the protective effects of rosiglitazone on corticosterone-induced injury (**Figures 7E,F**). Simultaneously, AV/PI was used for staining, and flow cytometry was used to analyze apoptotic astrocytes. The results showed that corticosterone induced early astrocytic apoptosis, and rosiglitazone could alleviate cellular apoptosis. This effect was reversed by T0070907 (**Figures 7G,H**). Rosiglitazone downregulated the expression of BAX, cleaved caspase 3, and cleaved PARP (PARP p85); this effect was abolished by T0070907 (**Figures 7I,J**). In sum, rosiglitazone protected the astrocytes of the primary cortex from corticosterone-induced apoptosis in a PPARγ-dependent manner.

**FIGURE 7:** Corticosterone-induced astrocyte apoptosis is relieved by rosiglitazone. **(A,B)** The vitality of astrocytes exposed to specific concentrations of corticosterone and rosiglitazone were measured by the MTT assay. **(C,D)** Western blotting analyzed the p-Akt/Akt of three astrocyte groups cultured in DMEM with or without IGF-1. **(E,F)** Hoechst labeled cells by immunofluorescence and quantified the number of astrocytes. **(G,H)** Flow cytometry measured the apoptosis of the corticosterone, rosiglitazone, and T0070907 (10 μM) groups. **(I,J)** The expression of apoptosis-associated proteins Bcl2 and BAX, total and cleaved caspase 3, and PARP were detected by WB. **(K–M)** The different IGF-1R and p-IRS1 expressions in astrocytes and neurons exposed to corticosterone, rosiglitazone, and T0070907 were detected by WB. **(N,O)** The ratios of p-Akt in whole-cell extracts and p-CREB in nucleoproteins differed under exposure to corticosterone, rosiglitazone, T0070907 (10 μM), and LY294002 (10 μM). Data are presented as means ± SEMs; *n* = 4–6 for all groups. ^∗^*p* < 0.05 vs. control, ^∗∗^*p* < 0.01 vs. control, ^∗∗∗^*p* < 0.001 vs. control, ^#^*p* < 0.05 vs. corticosterone, ^##^*p* < 0.01 vs. corticosterone, ^###^*p* < 0.001 vs. corticosterone, ^$^*p* < 0.05 vs. control, ^$$^*p* < 0.01 vs. control. cort, corticosterone; rosi, rosiglitazone; c+r, corticosterone + rosiglitazone; c+r+t, corticosterone + rosiglitazone+T007090; c+r+l, corticosterone + rosiglitazone+ LY294002.

As shown in **Figures 7C,D**, corticosterone significantly inhibited the phosphorylation of Akt in primary astrocytes compared with the control group, and rosiglitazone dramatically increased the p-Akt/Akt ratio. We also found that the IGF-1 receptor (IGF-1R) was more highly expressed in astrocytes than in neurons. Its substrate, insulin receptor substrate 1 (IRS-1), was phosphorylated when IGF-1 combined with IGF-1R (**Figures 7K–M**). Next, p-Akt/Akt expression in the cytoplasm and p-CREB/CREB expression in the cell nucleus were examined. Rosiglitazone was found to upregulate the phosphorylation of Akt and CREB, but this was inhibited by corticosterone. Both T0070907 and LY294002 (an Akt antagonist targeting PI3K) were found to inhibit the phosphorylation of Akt and CREB (**Figures 7N,O**). These findings indicate that rosiglitazone plays an anti-apoptotic role by acting on PPARγ and activating the Akt/CREB pathway.

### Rosiglitazone Improves Corticosterone-Induced Astrocytic Dysfunction, Thereby Protecting Cortex Neurons

Astrocytes are the most abundant glial cells in the brain. They play crucial roles in maintaining neuron function. In the present study, conditional medium from astrocytes exposed to corticosterone alone and corticosterone plus rosiglitazone was used to treat primary neurons, which mimicked the pharmacological environment *in vivo* (**Figure 8A**). The results showed that conditional medium from corticosterone-treated astrocytes increased the release of LDH from neurons, and this effect was reversed by conditional medium from corticosterone plus rosiglitazone-treated astrocytes (**Figure 8B**). Hoechst staining also showed that conditional medium from corticosterone plus rosiglitazone-treated astrocytes protected the neurons of the primary cortex from death (**Figure 8C**). Further, MAP2 antibodies were used to label the axons of the neurons. The results showed that neurons treated with conditional medium from corticosterone plus rosiglitazone-treated astrocytes had more and longer axons than neurons treated with conditional medium from corticosterone-treated astrocytes (**Figures 8D,E**).

**FIGURE 8:** Astrocyte supports neurons by secreting neurotrophic cytokines. **(A)** Astrocyte conditional medium was collected for culturing neurons. **(B)** The vitality of neurons exposed to conditional medium and specific concentrations of corticosterone or rosiglitazone was measured by detecting LDH secretion. **(C,D)** Immunofluorescence-labeled neurons and axons detected by Hoechst and MAP2. **(E)** The length of axons measured by ImageJ. (I) ACM. (II) ACM + rosiglitazone. (III) ACM + corticosterone. (IV) ACM + corticosterone + rosiglitazone. **(F)** Summary of the mechanism by which rosiglitazone relieves depression in astrocytes and neurons. Both autophagy and apoptosis ameliorated by rosiglitazone help maintain homeostasis in the mouse prefrontal cortex suffered CMS stimulation via specific pathway. Data are presented as means ± SEMs; *n* = 4 for LDH assay. ^∗^*p* < 0.05 vs. control, ^∗∗∗^*p* < 0.001 vs. control, ^###^*p* < 0.01 vs. corticosterone. cort, corticosterone; rosi, rosiglitazone; c+r, corticosterone + rosiglitazone.

## Discussion

Part of the difficulty in treating depression comes from the lack of any specific target that exerts effective long-term anti-depressive effects. PPARγ is a key regulator of metabolism and has been considered as a potential target for antidepressants. Rosiglitazone, a PPARγ agonist, has been reported to alleviate the depressive symptoms of patients with type 2 diabetes mellitus (Rasgon et al., 2010). The results of the present study show that mice subjected to UCMS exhibit depressive characteristics, including changes in weight and SPT values. Anhedonia, measured by decreases in SPT values, is the key indicator of depression in mice. In clinical settings, patients with depression have a tendency to lose body weight, and so do UCMS mice. FST and OFT indicate behavioral despair and social phobia, respectively. The results of the FST and OFT in our study provided evidence that UCMS mice e depressive or anxious behavior. These depressive behaviors were found to be alleviated by both rosiglitazone and fluoxetine, an effective antidepressant.

In addition to depressive behavior, depression is always accompanied by pathological changes such as inflammation, decreased neurogenesis and synaptic plasticity, and abnormal secretion of hormones or cytokines (Czeh et al., 2001; Cheng et al., 2014). The prefrontal cortex is an important part of the brain that modulates moods in both humans and rodents. Neuron or astrocyte dysfunction in the PFC is always involved in depression (Goldman-Rakic, 1996; Ma et al., 2016; Moreines et al., 2016). In our study, rosiglitazone relieved neural apoptosis in the PFC, as indicated by a TUNEL assay, and increased the number of GFAP-labeled astrocytes. Neuronal axons were improved by rosiglitazone, although the number of neurons was not significantly different. In fact, patients with depression exhibit little neuronal death, even though they show considerable neuronal dysfunction. It is well known that the extent of apoptosis and the survival conditions of astrocytes and neurons in the PFC influence mental disorders and diseases, including depression (Wen et al., 2015). The results of the present study indicate that rosiglitazone works as an antidepressant partly through its role in improving astrocyte and neuron function. Our *in vitro* results on astrocytes further confirmed the hypothesis that rosiglitazone protects astrocytes by inhibiting apoptosis.

A growing body of evidence suggests that inflammatory pathways are involved in the pathogeny of major depressive disorder and antidepressant response (Kalkman and Feuerbach, 2016; Wong et al., 2016). The antidepressant fluoxetine has been reported to affect inflammation (Alboni et al., 2016), and our study showed that rosiglitazone also reduces the levels of inflammation-related factors, including IL-6 and TNFα, in both mRNA and serum. Rosiglitazone has also been found to alleviate UCMS-induced abnormalities in the secretion of cytokines, such as IGF-1, CNTF, and NF-α1 (Thouennon et al., 2015). Elevation of the HPA axis is a common pathological feature of depression, and it can be activated via excessive secretion of glucocorticoid, thus exerting further negative effects on such targets as ovarian steroids, the gastrointestinal (GI) system, adipose tissue and its related peptides and microbiome, and the cardiovascular system (Duman et al., 2016). For rodents, the concentration of corticosterone increased significantly after UCMS modeling. This provided us with a method to investigate the mechanism by which rosiglitazone alleviated corticosterone stimulation of neurons and astrocytes *in vitro*. All of these findings illustrated that rosiglitazone alleviated depressive behavior in UCMS mice and exerted an antidepressant effect. However, the mechanism involved in rosiglitazone-mediated anti-depressive action remains unclear.

Autophagy is a ubiquitous phenomenon in eukaryocytes that plays a critical role in maintaining homeostasis and promoting cell survival (Yamamoto and Yue, 2014; Klionsky et al., 2016). Disorders of autophagy in the brain are responsible for various brain diseases, including depression (Abelaira et al., 2014; Gassen et al., 2014; Polajnar and Zerovnik, 2014; Jia and Le, 2015). The results of the present study showed elevated LC3B expression in PFC neurons, indicating increased autophagy in mice treated with rosiglitazone. Both *in vivo* and *in vitro*, rosiglitazone alleviated UCMS- and corticosterone-induced deficiencies in neuron autophagy. AMPK is a key metabolic kinase that can be phosphorylated at the Thr 172 site by several kinds of upstream kinases, including LKB1, TAK1, and CaMKKβ, and has been shown to influence depressive symptoms. Our *in vitro* results indicated that rosiglitazone upregulated the expression of LKB1 in neuron-like N2a-cell nuclei depending on PPARγ and thereby elevated the level of autophagy, which had been decreased by corticosterone stimulation. However, a recent study showed that rosiglitazone relieved mice of depressive behavior by inhibiting apoptosis but failed to affect autophagy (Patel et al., 2015). Yan et al. (2010) also reported that troglitazone could promote autophagy via activation of AMPKα. However, they found that troglitazone-mediated autophagy was independent of PPARγ, which was inconsistent with our results. In addition, the neuroprotective role of rosiglitazone via suppression of autophagic cell death has been reported in a global cerebral ischemia model (Shao and Liu, 2015). We believe that cell types and differences in stimuli may be responsible for the distinction. Taken together, these findings show that the regulation of autophagy by rosiglitazone plays important roles in several brain diseases.

Notably, rosiglitazone also showed a protective effect on astrocytes. PFC astrocytes suffered severe injury from UCMS, and this was attenuated by rosiglitazone. The modulation of corticosterone may constitute a link between *in vivo* CMS and *in vitro* stress, and corticosterone promotes apoptosis in the brain (Dumana et al., 1999). Our results showed an elevation of corticosterone and reduction of IGF-1 in the sera of UCMS mice. The hypothesis that rosiglitazone protects astrocytes from corticosterone-induced apoptosis was supported by the follow-up investigation. The main target of IGF-1, IGF-1R, was expressed more abundantly in primary astrocytes than in cortex neurons. The present study focused on astrocytes to investigate the manner by which the signal pathway mediated rosiglitazone’s effects. The results showed that rosiglitazone reversed corticosterone-induced IGF-1R and p-IRS1 reduction. Phosphorylated IRS1 activated the Akt/CREB pathway, thus playing the expected anti-apoptotic role. In this way, rosiglitazone increased the expression of IGF-1R in astrocytes by activating PPARγ.

In summary, rosiglitazone maintains the essential autophagy of neurons and N2a cells by elevating the expression of LKB1 and thus phosphorylating AMPK in the neurons of the prefrontal cortexes of mice. Moreover, rosiglitazone increases the concentration of IGF-1 in serum and the expression of IGF-1R in PFC astrocytes, thereby activating the Akt/CREB pathway and exerting an anti-apoptotic effect. Rosiglitazone also causes astrocytes to secrete neurotrophic cytokines and support neurons (**Figure 8F**). The crosstalk between astrocyte apoptosis and neuron autophagy remains to be assessed in future work, although we performed a preliminary exploration using the conditional medium from astrocytes to treat neurons. Overall, the present study revealed that rosiglitazone protects both neurons and astrocytes *in vivo* and *in vitro*, exerting an anti-depressive effect. These findings suggest that PPARγ may be a promising target for the development of antidepressants and may provide new insights for depression therapy.

## Author Contributions

X-LS conceived and designed the study, and drafting the manuscript. ZZ, LZ, and X-DG were responsible for all the *in vivo* experiments, qPCR assay and statistical analysis. ZZ, L-LC, T-FX, JY, and X-JZ performed immunohistochemistry and Western Blot assay. JJ and J-YH were responsible for the *in vitro* experiments. All authors reviewed the manuscript.

## Conflict of Interest Statement

The authors declare that the research was conducted in the absence of any commercial or financial relationships that could be construed as a potential conflict of interest.
